The article "Paricalcitol Attenuates Metabolic Syndrome-Associated Heart Failure through Enhanced Mitochondrial Fusion" was published in 2022. Journal: Oxid Med Cell Longev.

# Paricalcitol Attenuates Metabolic Syndrome-Associated Heart Failure through Enhanced Mitochondrial Fusion

**DOI:** 10.1155/2022/5554290

**Published:** 2022-06-11

**Authors:** Hina L. Nizami, Parmeshwar B. Katare, Pankaj Prabhakar, Ramu Adela, Soumalya Sarkar, Sudheer Arava, Praloy Chakraborty, Subir K. Maulik, Sanjay K. Banerjee

**Affiliations:** ^1^Non-Communicable Disease Group, Translational Health Science and Technology Institute (THSTI), Faridabad 121001, India; ^2^Department of Pharmacology, All India Institute of Medical Science (AIIMS), New Delhi 110029, India; ^3^Department of Endocrinology, All India Institute of Medical Science (AIIMS), New Delhi 110029, India; ^4^Department of Pathology, All India Institute of Medical Science (AIIMS), New Delhi 110029, India; ^5^Cardiology Department, VMMC and Safdarjung Hospital, New Delhi 110029, India; ^6^Department of Biotechnology, National Institute of Pharmaceutical Education and Research, Guwahati 781101, India

## Abstract

**Objectives:**

Transition from cardiac hypertrophy to failure involves adverse metabolic reprogramming involving mitochondrial dysfunction. We have earlier shown that vitamin D deficiency induces heart failure, at least in part, through insulin resistance. However, whether activation of vitamin D receptor (VDR) can attenuate heart failure and underlying metabolic phenotype requires investigation. Thus, we aimed to assess the cardioprotective potential of paricalcitol, a vitamin D receptor-activator, against cardiac hypertrophy and failure in high-fat high-fructose-fed rats.

**Methods:**

Male Sprague Dawley rats were fed control (Con) or high-fat high-fructose (HFHFrD) diet for 20 weeks. After 12 weeks, rats from HFHFrD group were divided into the following: HFHFrD, HFHFrD+P (paricalcitol *i.p.* 0.08 *μ*g/kg/day) and HFHFrD+E (enalapril maleate *i.p.* 10 mg/kg/day). Intraperitoneal glucose tolerance test, blood pressure measurement, and 2D echocardiography were performed. Cardiac fibrosis was assessed by Masson's trichrome staining of paraffin-embedded heart sections. Mitochondrial DNA and proteins, and citrate synthase activity were measured in rat hearts. VDR was silenced in H9c2 cardiomyoblasts, and immunoblotting was performed.

**Results:**

Paricalcitol improved glucose tolerance, serum lipid profile, and blood pressure in high-fat high-fructose-fed rats. Paricalcitol reduced cardiac wall thickness and increased ejection fraction in high-fat high-fructose-fed rats but had no effect on perivascular fibrosis. PGC1-*α* was upregulated in the HFHFrD+P group compared to the HFHFrD group, but there was no significant difference in mitochondrial content. Citrate synthase activity was significantly higher in the HFHFrD+P group compared to the HFHFrD group. Rat hearts of the HFHFrD+P group had significantly higher expression of mitofusins. H9c2 cells with VDR knockdown showed significantly lower expression of Mfn2. Improvement in the HFHFrD+P group was comparable with that in the HFHFrD+E group.

**Conclusions:**

Paricalcitol reverses cardiac dysfunction in rats with metabolic syndrome by enhancing mitochondrial fusion. We demonstrate repurposing potential of the drug currently used in end-stage kidney disease.

## 1. Introduction

Heart failure is a public health problem with persistently rising prevalence due to increase in ageing population [1]. Maladaptive cardiac remodeling, in response to injury or comorbid conditions such as diabetes and hypertension, and ventricular dilatation, and impaired contractility constitute systolic heart failure [2]. Its diagnosis is clinically confirmed by echocardiographic observation of impaired myocardial and valvular structure and function. Treatment options include pharmacologic therapy, implantable devices, lifestyle changes, and surgery. Drug therapy is mainly aimed at relief of symptoms (e.g., diuretics) and improvement of residual cardiac function (e.g., ACE inhibitors, beta blockers, and aldosterone antagonists). Heart failure often coexists with other morbidities such as metabolic syndrome, renal impairment, and anemia, which further complicates the treatment.

We have earlier shown vitamin D deficiency is associated with increased prevalence of type 2 diabetes both with and without coexisting coronary artery disease, both important risk factors for heart failure [3]. We have also demonstrated the role of vitamin D deficiency as an independent risk factor for cardiac hypertrophy and heart failure in rats, through induction of myocardial insulin resistance [4]. In experimental and clinical studies, respectively, VDR knockdown or vitamin D deficiency is associated with remarkable cardiac hypertrophy, activation of the renin angiotensin system, cardiac dysfunction, and failure [5, 6]. However, experimental and clinical reports of vitamin D supplementation yield contradicting data about possible benefits [7, 8]. Reduced activation of vitamin D due to hepatic or renal dysfunction and sequestering of vitamin D in fat stores in obesity are some possible reasons for the loss of beneficial effects in disease, and hence, synthetic, nonhypercalcemic analogues might be preferable alternatives [9, 10]. Paricalcitol is an FDA-approved drug used in the management of end-stage kidney disease and has shown cardiorenal benefits in various experimental models [11, 12].

Though heart failure is essentially a decompensated state of cardiac muscle contractility, it is also marked by deficits in cardiac bioenergetics. Energy transduction in the heart depends majorly on oxidative phosphorylation in the mitochondria; excessive fatty acid oxidation in the absence of glucose leads to respiratory uncoupling and oxidative stress [13]. Mitochondrial dynamics are under control of processes such as fusion, fission, and biogenesis, and insulin is known to directly promote mitochondrial fusion through optic atrophy protein 1 (OPA1) [14]. Myocardial insulin resistance and mitochondrial dysfunction have been shown to be involved in the transition of heart from diastolic dysfunction to systolic failure in a model of pressure overload-hypertrophy in rats [15]. Successful use of therapies such as trimetazidine, omega-3 fatty acid, and perhexiline indicates that metabolic modulation might be an attractive therapeutic strategy to manage the development and progression of heart failure [16, 17].

Vitamin D receptor is a nuclear receptor conventionally known to be involved in transcription of target genes involved in calcium absorption and bone formation. However, the pleiotropic extraskeletal effects of VDR are under investigation in various tissues [18, 19]. Vitamin D has been shown to favourably affect metabolic functions such as insulin signalling and lipid metabolism in both experimental and clinical samples [20–22]. High circulating level of free fatty acidscan contribute to both insulin resistance and mitochondrial dysfunction. Regulation of mitochondrial structure, content, and bioenergetics by 1,25-OH vitamin D3 has been reported in peripheral blood mononuclear cells, adipocytes, skeletal muscle, and various cancer cell lines [23–26]. In homocysteine-treated rat heart slices, treatment with vitamin D3 improved mitochondrial function and redox status [27]. However, the possible effect of VDR modulation on myocardial mitochondrial dynamics in metabolic syndrome-associated cardiac failure requires investigation.

We aimed to investigate the therapeutic potential of paricalcitol in cardiac dysfunction in rats with metabolic syndrome, through its possible effect on cardiac mitochondrial dynamics. Animals were fed high-fat high-fructose diet and treated with paricalcitol, and cardiometabolic outcomes were assessed. Since renin angiotensin system blockade has known clinical benefit against cardiac remodeling and failure, enalapril was used as the standard therapy in a group of high-fat high-fructose fed rats.

## 2. Research Designs and Methods

### 2.1. Animals

Male Sprague Dawley rats (200-220 g) were procured from All India Institute of Medical Sciences, New Delhi, and maintained in Small Animal facility of THSTI, Faridabad. Rats were provided food and water *ad libitum* throughout the study period, with the exception of the 12-hour fasting period preceding blood sample withdrawal and intraperitoneal glucose tolerance test. All experimental procedures involving animals were performed according to the relevant regulations and guidelines of Institutional Animal Ethical Committee (IAEC) of Translational Health Science and Technology Institute, Faridabad (IAEC/THSTI/2015-3).

### 2.2. Materials

Paricalcitol was purchased from Cayman Chemical Company (#17716). Enalapril maleate was procured from LKT Labs (#E5201). Antibodies against VDR (ab3508; 1 : 500), PGC1-*α* (ab54481; 1 : 1000), MFN1 (ab57602; 1 : 1000), and MFN2 (ab137037; 1 : 1000) were purchased from Abcam.

### 2.3. In Vivo Study Design and Drug Treatment

Control (65% corn starch diet; Cat. No. D11708B) and high-fat high-fructose (45% kcal% fat and 35% kcal% fructose; Cat. No. D08040105G) diets were purchased from Research Diets, USA. After an acclimatization period of one week, rats were randomized into two groups and were fed either control diet (CON) or high-fat high-fructose diet (HFHFrD) for 20 weeks. At the end of 12 weeks, intraperitoneal glucose tolerance test and echocardiography were performed, and rats from the HFHFrD group were further divided into three groups: HFHFrD, HFHFrD+P (paricalcitol *i.p.* 0.08 *μ*g/kg/day), and HFHFrD+E (enalapril maleate *i.p.* 10 mg/kg/day). The experimental design is illustrated in Figure 1. At the end of the remaining 8 weeks, rats from all the groups were sacrificed; serum samples and heart tissues were collected and stored at a -80°C refrigerator for further analysis. Experimental methods have been adapted from our previously published work [4].

### 2.4. Intraperitoneal Glucose Tolerance Test

At the end of 12 and 20 weeks, after an overnight fasting period, rats were given an intraperitoneal bolus injection of glucose (2 g/kg *BW*). Blood glucose sampling was performed at 0 (just before), 15, 30, 60, and 120 minutes post glucose administration, using a commercially available blood glucose measurement system (OneTouch Select Plus, Johnson & Johnson).

### 2.5. Serum Biochemistry

Insulin (Crystal Chem, USA), triglycerides (BioVision, USA), HDL cholesterol (BioVision, USA), and free fatty acids (BioVision, USA) were measured in rat serum samples using commercially available assay kits.

### 2.6. Noninvasive Blood Pressure Measurement

Blood pressure was evaluated at the end of the study (20 weeks) using the Non-Invasive Blood Pressure System (Harvard Apparatus), complying with manufacturer's protocol. Animals were trained daily in restrainers for 4 days prior to experimental data recording. To record blood pressure, a tail cuff and sensor were placed about 2 cm from the tip of the animal's tail, and blood pressure was recorded. Five individual measurements were made and analysed as mean for each animal.

### 2.7. Echocardiography

Echocardiography was performed after the completion of 12 and 20 weeks. Rats were anesthetized using a cocktail of ketamine (80 mg/kg BW *i.p.*) and xylazine (8 mg/kg BW *i.p.*). Two-dimensional and M-mode echocardiograms were obtained using a fully digitized instrument (HD11 XE, Philips) with a hand-held 12 MHz neonatal cardiac probe transducer placed at a short axis view at the level of the papillary muscles of the left ventricle. Diastolic left ventricular posterior wall (LVPW) and intraventricular septum (IVS) thicknesses were recorded. Left ventricular internal diastolic dimension (LVIDd) and LV internal systolic dimension (LVIDs) were also recorded. Fractional shortening and ejection fraction values were derived from the dimensions recorded above. Image acquisition and analysis were performed by an analyst blind to the experimental groups.

### 2.8. Cardiac Hypertrophy Measurement

Heart weight-to-tail length ratio of rats was used to evaluate cardiac hypertrophy. Briefly, at the end of 20 weeks, animals from all groups were sacrificed, hearts were isolated, rinsed in ice-cold PBS, and blotted, and their weight was measured. The ratio of heart weight and tail length was calculated and expressed in gcm^−1^.

### 2.9. Histopathology

At the end of 20 weeks, the heart tissue was harvested and fixed in phosphate-buffered formalin (10%). Fixed samples were embedded in paraffin and sectioned for histopathological analysis. Sections of 5 *μ*m thickness were stained with haematoxylin-eosin (H&E) and Masson's trichrome stains and examined under a light microscope.

### 2.10. Mitochondrial Content/Mass Measurement

Mitochondrial mass/content was estimated by analysing mitochondrial DNA expression and normalising it to nuclear DNA expression. DNA was isolated from rat hearts using the GF1-Tissue/Blood FNA Extraction kit (Vivantis) as per manufacturer's protocol. DNA concentration and quality were measured using NanoDrop spectrophotometer (Thermo Scientific). Polymerase chain reaction (PCR) was set up using EmeraldAmp PCR Mastermix (Takara, USA) on Veriti Thermal Cycler (Applied Biosystems). Nuclear beta 2-microglobin expression was used as a reference to normalise the mitochondrial CO-1 (cytochrome oxidase C subunit 1) expression data. Primer sequences are listed in Table 1.

### 2.11. Cell Culture

H9c2 cells, purchased from ATCC (USA), were cultured in DMEM supplemented with 10% FBS, at 37°C in a 5% CO_2_ incubator. VDR was silenced by transfecting H9c2 cells with shRNA against VDR (Origene) using Xtremgene HP Transfection Reagent (Roche), and transfected cells were used to establish a stable cell line using puromycin as a selecting agent.

### 2.12. Western Blotting

Rat heart tissues and H9c2 cells were lysed in ice-cold RIPA buffer (Pierce) and were then centrifuged at 12000 rpm for 20 minutes at 4°C. Bicinchoninic acid (BCA) assay (Thermo Scientific) was used to measure protein content. Proteins (30 *μ*g) were resolved on 10-12% SDS-polyacrylamide gel using TGX stain free kit (Bio-Rad). After electrophoresis, proteins were blotted on to polyvinylidine difluoride (PVDF) membrane (Merck Millipore). Membrane was blocked in 3% nonfat dry milk in TBST (0.1% Tween 20) or 5% BSA solution at room temperature for an hour, followed by incubation with desired primary antibody overnight at 4°C. After three washes with TBST, the membrane was incubated with the appropriate HRP-labeled secondary antibody at room temperature for an hour. Membrane was washed with TBST (thrice for 5 min each), and the blot was visualized using Gel Doc XR system (Bio-Rad), using Roche Lumi Light substrates (Thermo Scientific). Protein expression was normalised to corresponding stain free gel (BioRad™) loading controls' expression.

## 3. Results

### 3.1. Paricalcitol Improves Glucose Tolerance in High-Fat High-Fructose-Fed Rats

#### 3.1.1. Fasting Blood Glucose and Serum Insulin

There was a significant increase in fasting blood glucose of HFHFrD group as compared to that of the Con group, at the end of 20 weeks (Figure 2(a)). However, we did not observe any significant difference in the HFHFrD+P and HFHFrD+E groups, in comparison to the HFHFrD group (Figure 2(a)).

Similarly, there was a significant increase in fasting serum insulin of the HFHFrD group as compared to the Con group (Figure 2(b)). However, no significant difference was observed in the HFHFrD+P and HFHFrD+E groups, in comparison to the HFHFrD group (Figure 2(b)).

#### 3.1.2. HOMA Analysis

At the end of twenty weeks, HOMA-IR of the HFHFrD group was significantly higher than that of the Con group (Figure 2(c)). However, no significant difference was observed in the HFHFrD+P and HFHFrD+E groups, in comparison to the HFHFrD group (Figure 2(c)).

No significant difference was found between HOMA-B values of different groups (Figure 2(d)).

#### 3.1.3. Intraperitoneal Glucose Tolerance Test

In the intraperitoneal glucose tolerance test (IPGTT) performed at the end of 12 weeks, the HFHFrD group showed raised blood glucose time-profile and significantly higher area-under-curve (AUC) than the Con group (Figure 2(e)), indicating impaired blood glucose disposal in these rats.

In the IPGTT performed at the end of 20 weeks, the HFHFrD group showed impaired glucose tolerance and higher area under curve, compared to the Con group (Figures 2(f) and 2(g)). After 8 weeks of treatment with paricalcitol, the HFHFrD+P group showed significantly improved glucose tolerance in IPGTT, with significantly lower area under curve, compared to the HFHFrD group (Figures 2(f) and 2(g)).

### 3.2. Paricalcitol Attenuates Dyslipidemia in High-Fat High-Fructose-Fed Rats

We observed significantly higher serum triglycerides and free fatty acids in the HFHFrD group compared to the Con group (Figures 3(a) and 3(b)). After 8 weeks of treatment with paricalcitol, the HFHFrD+P group showed significantly decreased triglycerides and free fatty acids, compared to the HFHFrD group (Figures 3(a) and 3(b)). The HFHFrD+E group showed significant decrease in serum free fatty acids, compared to the HFHFrD group (Figure 3(b)). There were no significant changes in serum HDL cholesterol in the different groups (Figure 3(c)).

### 3.3. Paricalcitol Attenuates Hypertension in High-Fat High-Fructose-Fed Rats

There were significant increases in systolic, diastolic, and mean arterial blood pressure in the HFHFrD group, compared to the Con group (Figures 3(d)–3(f)). After 8 weeks of treatment with paricalcitol or enalapril, the HFHFrD+P group showed significantly decreased blood pressure, compared to the HFHFrD group (Figures 3(d)–3(f)).

### 3.4. Paricalcitol Attenuates Cardiac Hypertrophy in High-Fat High-Fructose-Fed Rats

At the end of 20 weeks, we observed significant increase in the heart weight-to-tail length ratio in the HFHFrD group, when compared to the Con group (Figure 3(g). After treatment with paricalcitol for 8 weeks, the HFHFrD+P and HFHFrD+E groups showed significant decrease in heart weight-to-tail length, as compared to the HFHFrD group (Figure 3(g)).

### 3.5. Paricalcitol Attenuates Left Ventricular Hypertrophy and Systolic Dysfunction in High-Fat High-Fructose-Fed Rats

#### 3.5.1. Cardiac Wall Thickness

To study changes in the cardiac structure and function, we performed 2D echocardiography at the end of 12 and 20 weeks. At the end of 20 weeks, there was a significant increase in the intraventricular septum thickness (IVSd) and left ventricular posterior wall thickness (LVPWd) in the HFHFrD group, compared to the control group (Figures 4(a) and 4(b)). The HFHFrD+P and HFHFrD+E groups had significantly decreased IVSd and LVPWd compared to the HFHFrD group, at the end of 20 weeks. Also, IVSd had significantly decreased in the HFHFrD+P and HFHFrD+E groups between 12 and 20 weeks, indicating curative effect of the treatment with paricalcitol and enalapril (Figures 4(a) and 4(b)).

#### 3.5.2. Cardiac Chamber Diameters

We did not observe significant changes in the diastolic left ventricular internal diameter (LVIDd) (Figure 4(c)). However, there was a significant increase in the systolic left ventricular internal diameter (LVIDs) of the HFHFrD group compared to the Con group, at the end of 20 weeks (Figure 4(d)). This indicated dilatation of the left ventricle in the HFHFrD group. The HFHFrD+P and HFHFrD+E groups showed significant decrease in LVIDs compared to the HFHFrD group, at the end of 20 weeks. Also, LVIDs showed significant decrease in the HFHFrD+P group between 12 and 20 weeks, indicating curative effect of the treatment with paricalcitol (Figure 4(d)).

#### 3.5.3. Cardiac Contractile Function

At the end of 20 weeks, there was a significant decrease in the fractional shortening (FS) and ejection fraction (EF) in the HFHFrD group, compared to the control group (Figures 4(e) and 4(f)). The HFHFrD+P and HFHFrD+E groups significantly improved in FS and EF compared to the HFHFrD group, at the end of 20 weeks. Also, FS significantly improved in the HFHFrD+P and HFHFrD+E groups between 12 and 20 weeks, indicating curative effect of the treatment with paricalcitol and enalapril (Figure 4(e)).

### 3.6. Paricalcitol Does Not Affect Myocardial Fibrosis in High-Fat High-Fructose-Fed Rats

We observed no significant differences in histopathological features among the different groups based on haematoxylin and eosin (H&E)-stained rat heart sections (Figure 5(a)). In the Masson trichrome stained heart sections, increased perivascular fibrosis was observed in the HFHFrD group (Figure 5(b)). However, no significant improvement was observed in the HFHFrD+P and HFHFrD+E groups, compared to the HFHFrD group (Figure 5(b)).

### 3.7. Paricalcitol Increases Cardiac PGC1-*α* Expression in High-Fat High-Fructose-Fed Rats

PGC1-*α* induces mitochondrial biogenesis through activation of transcription factors such as NRF-1 and NRF-2. At the end of the study, PGC1-*α* expression was lower in the HFHFrD group, compared to the Control group, though not statistically significant (Figure 6(b)). Treatment with paricalcitol caused significantly higher expression of PGC1-*α* protein in the HFHFrD+P group, compared to the HFHFrD group. The enalapril also significantly upregulated PGC1-*α* expression, similar to paricalcitol (Figure 6(b)).

### 3.8. Paricalcitol Does Not Alter Mitochondrial Mass/Content in High-Fat High-Fructose-Fed Rats

Since we observed increased expression of PGC1-*α* expression in the hearts of the HFHFrD+P group, we evaluated the effect of paricalcitol on mitochondrial mass/content. Change in mitochondrial DNA content is a marker of changing mitochondrial mass. We observed no significant differences in mitochondrial DNA/content between the different experimental groups, calculated from the expression of mitochondrial CO-1 normalised to beta 2-microglobin (Figure 6(d)).

### 3.9. Paricalcitol Increases Cardiac Citrate Synthase Activity in High-Fat High-Fructose-Fed Rats

At the end of the study, we evaluated citrate synthase activity in the rat hearts. It was significantly lower in the HFHFrD group, compared to the Con group (Figure 6(e)). Treatment with paricalcitol, but not with enalapril, significantly increased citrate synthase activity in the HFHFrD+P group, compared to the HFHFrD group.

### 3.10. Paricalcitol Increases Cardiac Expression of Mfn2 in High-Fat High-Fructose-Fed Rats

Since we observed an increase in citrate synthase activity with paricalcitol treatment, we next studied the expression of Mfn1 and Mfn2 that are involved in mitochondrial fusion. There was no significant change in the expression of Mfn1 and Mfn2 in the HFHFrD group compared to the Con group (Figure 7(b)). The increase in Mfn1 expression in both the HFHFrD+P and HFHFrD+E groups was not significant, compared to the HFHFrD group. Paricalcitol and enalapril significantly increased the expression of Mfn2 in the HFHFrD+P group, compared to the HFHFrD group (Figure 7(c)).

### 3.11. VDR Knockdown Causes Downregulation of Mfn2 in H9c2 Cardiomyoblasts

Since paricalcitol upregulated the expression of Mfn2 in a high-fat high-fructose-fed rat heart, we next investigated whether VDR is directly involved in the regulation of cardiac expression of mitofusins. We observed that VDR silencing in H9c2 cardiomyoblasts causes a significant decrease in Mfn2 expression, but not in Mfn1 expression (Figures 7(e) and 7(f)).

## 4. Discussion

Vitamin D has been gaining attention for nonclassical roles such as regulation of inflammation, immunity, cell cycle, and metabolism. Association between vitamin D deficiency and adverse cardiometabolic outcomes has been repeatedly shown in patients, but the therapeutic role of vitamin D supplementation remains controversial [3, 28, 29]. Clinical studies have yielded conflicting results regarding the potential benefits of vitamin D in subjects with cardiometabolic diseases [30, 31]. In view of reduced bioavailability of the active form of vitamin D in disease conditions, use of vitamin D analogues such as paricalcitol and maxacalcitol has been investigated [32]. Paricalcitol has shown therapeutic benefit in experimental models of kidney disease, diabetes, and their cardiovascular complications [33, 34]. However, its effect on metabolic syndrome-associated heart failure remained to be investigated. In this study, we have demonstrated the cardioprotective effects of paricalcitol treatment in a high-fat high-fructose-fed rat model of metabolic syndrome.

Rats were fed diets with high fat and high fructose to induce metabolic syndrome. Hypercaloric diets containing high fat and high fructose have been shown to induce hyperinsulinemia and impaired glucose tolerance [35]. Insulin resistance is considered a principal component of diet-induced metabolic syndrome [36, 37]. In our study, animals of the HFHFrD group showed elevated blood glucose, serum insulin, and HOMA-IR values, indicating development of a prediabetes-like state. Treatment with paricalcitol for 8 weeks did not cause any significant changes in these parameters. However, paricalcitol reversed the impairment of blood glucose disposal in the intraperitoneal glucose tolerance test in the HFHFrD+P group.

High-calorie diets are known to disturb serum lipid profile with an increase in serum triglycerides and free fatty acids [38]. In this study, we observed increase in triglycerides and free fatty acids in serum of rats in the HFHFrD group. Treatment with paricalcitol attenuated these changes and improved lipid profile of the HFHFrD+P group. No significant differences were observed in the HDL cholesterol levels of the different groups. The lipid-lowering effect of paricalcitol in metabolic syndrome has not been reported earlier.

Apart from triggering metabolic derangements such as insulin resistance and dyslipidemia, high-fat high-fructose diet also causes cardiovascular perturbations [35]. At the end of the study, we observed raised systolic, diastolic, and mean arterial blood pressure in the HFHFrD group. Treatment with paricalcitol significantly reduced blood pressure in the HFHFrD+P group. Hypertension is an established predictor of cardiac hypertrophy, due to resultant increase in cardiac workload. Heart weight-to-tail length ratio, an index of cardiac size, was increased significantly in the HFHFrD group compared to the Con group. Treatment with paricalcitol was associated with a significant decrease in heart weight-to-tail length ratio in the HFHFrD+P group. Similar to our findings, paricalcitol has earlier been shown to attenuate cardiac hypertrophy in experimental models of pressure overload, hypertension, and uremia [39–41].

As a consequence of its metabolic effects, high-fat high-fructose diet also induces cardiac remodeling [35]. At the end of 20 weeks, there was significant increase in the intraventricular septum and left ventricular posterior wall thicknesses in the HFHFrD rats. We observed significant decrease in cardiac wall thicknesses in the HFHFrD+P group, indicating attenuation of cardiac hypertrophy. Though initially an adaptive response, unmitigated left ventricular hypertrophy progresses to cardiac failure. Metabolic syndrome is known to increase the risk of left ventricular systolic dysfunction by two folds [42]. Echocardiography is considered the gold-standard diagnostic technique for systolic failure; hence, we used it to assess systolic function in these rats. In the HFHFrD rats, we observed increased systolic internal dimension of the left ventricle, indicating dilatation and systolic dysfunction. This led to significantly reduced fractional shortening and ejection fraction, which implies compromised cardiac contractility. In the HFHFrD+P group, systolic function was markedly improved. According to earlier studies, paricalcitol prevents the progression of hypertrophy to heart failure in Dahl salt-sensitive hypertensive rats [40].

Interestingly, paricalcitol did not only attenuate the high-fat high-fructose-induced cardiac perturbations seen at the end of 20 weeks, it also reversed the progression of cardiac dysfunction induced by high-fat high-fructose diet seen at the end of 12 weeks. The improvement in systolic function is an interesting finding because the current treatment regimens for heart failure only manage the symptoms and do not reverse cardiac dysfunction. An important underlying pathology here is the pathological remodeling of the heart. Increased cardiac load due to factors such as hypertension, sympathetic tone, and others can trigger reactive myocardial fibrosis [43]. These fibrotic changes usually begin in the perivascular region and slowly spread into the myocardium. Perivascular fibrosis was observed in the HFHFrD group through observation of Masson's trichrome-stained heart sections. We speculated that attenuation or reversal of this fibrosis might be responsible for cardioprotective effect of paricalcitol, seen earlier. However, we did not observe any significant difference in the HFHFrD+P group, as compared to the HFHFrD group. This is similar to earlier reports where paricalcitol had no protective effect on perivascular fibrosis in rats with renal insufficiency and low vitamin D [44]. These findings warranted further investigation into the factors underlying the protective effect of paricalcitol in high-fat high-fructose-induced cardiac dysfunction.

Since there were no significant improvements in cardiac structure or remodelling status and functional improvements were observed, it indicated improvement in the functional status of the cardiac muscle. The myocardium relies on continuous supply of ATP to sustain its contractility. Mitochondria are the cellular organelles that generate the required ATP for energy transduction in heart. Defects in structure, function, or dynamics of mitochondria adversely affect cardiac function. Mitochondrial dysfunction has been shown to underlie progression of cardiac hypertrophy to heart failure [45]. Hypercaloric diets can cause mitochondrial dysfunction through increased flux of fats and glucose [46]. Mitochondrial biogenesis, which implies formation of new mitochondria, might be impaired in conditions of unmitigated stress [44]. In our study also, we observed that expression of PGC1-*α* was downregulated in HFHFrD rat hearts. PGC1-*α* drives mitochondrial biogenesis through activation of downstream transcription factors [47, 48]. In the HFHFrD+P group, increased expression of PGC1-*α* was observed. In earlier reports, vitamin D supplementation has been shown to upregulate PGC1-*α* expression in rat skeletal muscle [49].

Increased cardiac expression of PGC1-*α* after paricalcitol treatment led us to speculate an increase in mitochondrial mass/content in the HFHFrD group. Mitochondrial mass/content can be quantified using mitochondria-tagging fluorescent dyes or by measuring mitochondrial DNA amount. We measured the expression of CO-1 gene that is encoded in mitochondrial DNA and normalised it to expression of beta 2-microbin encoded in nuclear DNA. Surprisingly, we did not observe any significant changes between the fold changes of CO-1 expression between different groups. This indicated that there was no significant increase in mitochondrial content in HFHFrD+P rat hearts, despite upregulation of PGC1-*α*. This could be due to regulation of PGC1-*α* function by posttranslational modifications. However, activity of myocardial citrate synthase improved in the HFHFrD+P group, compared to the HFHFrD group. Acetyl CoA generated from glycolysis and fatty acid oxidation enters Kreb's cycle in the mitochondrial matrix. Citrate synthase is the first enzyme of this biochemical cycle, and its activity is thus considered a hallmark of mitochondrial health [50]. Our findings indicate that paricalcitol improves mitochondrial function in high-fat high-fructose-fed rats.

Our next question was how mitochondrial function could improve without any changes in mitochondrial content or biogenesis. Mitochondrial dynamics are controlled not only through biogenesis but also through fusion and fission. Mitochondrial fusion improves mitochondrial function by fusing of healthy mitochondrial fractions and recycling of damaged components [51]. We examined the expression of mitofusins (Mfn2) that are the proteins involved in mitochondrial fusion. Myocardial expression of Mfn2 increased significantly in the HFHFrD+P group, compared to the HFHFrD group. Mfn2 has been earlier described as a therapeutic target for diabetic cardiomyopathy through inhibition of mitochondrial fission in db/db mice [52]. It has also been shown to be protective against angiotensin-mediated cardiomyocyte injury by induction of mitophagy and mitochondrial fusion [48].

The findings above indicate that paricalcitol improved mitochondrial function, possibly through improvement of mitochondrial dynamics. To confirm that this beneficial effect was mediated by activation of VDR by paricalcitol, we performed further experiments *in vitro*. To perform loss-of-function studies regarding the effect of VDR on mitochondrial fusion, we silenced VDR in H9c2 cardiomyoblasts. Here, we observed that the expression of Mfn2, but not Mfn1, was remarkably reduced in H9c2 cells with VDR knockdown.

## 5. Summary and Conclusion

In this study, we demonstrate that paricalcitol, a vitamin D receptor activator, attenuates metabolic syndrome-associated cardiac dysfunction in rats. High-fat high-fructose diet induces glucose intolerance, dyslipidemia, hypertension, fibrosis, and cardiac dysfunction in rats. Paricalcitol improves glucose tolerance, lipid profile, blood pressure, and cardiac contractility, but does not attenuate myocardial fibrosis. We demonstrate that the VDR activator paricalcitol improves cardiometabolic function in rats, possibly through improvement of mitochondrial dynamics. Despite increase in cardiac PGC1-*α* expression, change in mitochondrial content is not observed in paricalcitol-treated rats with metabolic syndrome. However, paricalcitol-induced increase in citrate cynthase activity and expression of Mfn2 indicates the possible role of VDR activation in mitochondrial fusion. Further investigation is warranted into the detailed mechanism of activation of Mfn2 and its effect on other mitochondrial function parameters. Decreased expression of mitofusin 2 in VDR-silenced H9c2 cells provided evidence about the positive role of VDR in mitochondrial fusion. These findings indicate potential for repurposing of paricalcitol for treatment of cardiac failure associated with conditions such as prediabetes and diabetes mellitus.

## Figures and Tables

**Figure 1:** Schematic representation of experimental animal study design.

**Figure 2:** Paricalcitol improves glucose tolerance in high-fat high-fructose-fed rats. (a) Fasting blood glucose. (b) Fasting serum insulin. (c) HOMA IR. (d) HOMA-B. (e) Intraperitoneal glucose tolerance test (12 weeks). (f) Intraperitoneal glucose tolerance test (20 weeks). (g) Area under the curve (20 weeks IPGTT). Data expressed as mean ± SEM (*n* = 6). ^∗^*p* < 0.05,  ^∗∗^*p* < 0.01, and^∗∗∗^*p* < 0.001 vs. the Con group. ^#^*p* < 0.05 vs. the HFHFrD group.

**Figure 3:** Paricalcitol attenuates dyslipidemia, hypertension and cardiac hypertrophy in high-fat high-fructose-fed rats. (a) Serum triglycerides. (b) Serum free fatty acids. (c) Serum HDL cholesterol. (d) Systolic blood pressure. (e) Diastolic blood pressure. (f) Mean arterial pressure. (g) Heart weight/tail length ratio. Data expressed as mean ± SEM (*n* = 6). ^∗^*p* < 0.05 and^∗∗^*p* < 0.01 vs. the CON group, ^#^*p* < 0.05, ^##^*p* < 0.01, and ^###^*p* < 0.001 vs. the HFHFrD group.

**Figure 4:** Paricalcitol reverses cardiac hypertrophy and failure in high-fat high-fructose-fed rats. (a) Intraventricular septum thickness (diastole). (b) Left ventricular posterior wall thickness (diastole). (c) Left ventricular internal dimension (diastolic). (d) Left ventricular internal dimension (systolic). (e) Fractional shortening. (f) Ejection fraction. Data expressed as mean ± SEM (*n* = 4-5). ^∗^*p* < 0.05 and^∗∗∗^*p* < 0.001 vs. the CON group. ^#^*p* < 0.05, ^##^*p* < 0.01, and ^###^*p* < 0.001 vs. the HFHFrD group.

**Figure 5:** Paricalcitol does not affect myocardial fibrosis in high-fat high-fructose-fed rats. (a) Representative micrograph of haematoxylin and eosin-stained rat heart sections. (b) Representative micrograph of Masson's trichrome-stained rat heart sections.

**Figure 6:** Paricalcitol does not alter myocardial mitochondrial content in high-fat high-fructose-fed rats. (a) Representative western blot image of PGC1-*α*. (b) Densitometry analysis of PGC1-*α* expression. (c) Representative agarose gel image of CO-1 and beta 2-microglobin PCR products. (d) Densitometry analysis of CO-1 expression. (e) Fold change in citrate synthase activity. Protein expression data were normalised to the expression of stain free gel (TGX Stain-FreeTM FastCastTM BioRadTM) image. ^##^*p* < 0.01 vs. HFHFrD group. CO-1 expression data were normalised to beta 2-microglobin expression. Data expressed as mean ± SEM (*n* = 3 for Western blot and agarose gel electrophoresis; *n* = 5 for citrate synthase activity). ^∗^*p* < 0.05 vs. Control; ^##^*p* < 0.01 vs. HFHFrD.

**Figure 7:** Vitamin D receptor modulates myocardial expression of mitofusin 2. (a) Representative western blot images of Mfn1 and Mfn2 in rat hearts. (b) Densitometry analysis of Mfn1 expression in rat hearts. (c) Densitometry analysis of Mfn2 expression in rat hearts. (d) Representative western blot images of VDR, Mfn1, and Mfn 2 in H9c2 cells. (e) Densitometry analysis of Mfn1 in H9c2 cells. (f) Densitometry analysis of Mfn2 in H9c2 cells. Protein expression data were normalised to the expression of stain free gel (TGX Stain-FreeTM FastCastTM BioRadTM) image. Data expressed as mean ± SEM (*n* = 3). ^∗^*p* < 0.05 vs. the Control group; ^∗∗∗^*p* < 0.001 vs. the Control group.

**Table 1:** List of primers used in mitochondrial content measurement.

Gene	Forward primer	Reverse primer
CO-1	CACATGAGCAAAAGCCCACT	ACGGCCGTAAGTGAGATGAA
Beta 2-microglobin	GATCACTTGTCCGGAGTAGAA	ACGTAGCAGTTGAGGAAGTTG

## Data Availability

Data are available upon reasonable request.

## References

[1] Conrad N., Judge A., Tran J. (2018). Temporal trends and patterns in heart failure incidence: a population-based study of 4 million individuals. *The Lancet*.

[2] McMurray J. J. (2010). Systolic heart failure. *New England Journal of Medicine*.

[3] Adela R., Borkar R. M., Bhandi M. M. (2016). Lower vitamin D metabolites levels were associated with increased coronary artery diseases in type 2 diabetes patients in India. *Scientific Reports*.

[4] Nizami H. L., Katare P., Prabhakar P. (2019). Vitamin D deficiency in rats causes cardiac dysfunction by inducing myocardial insulin resistance. *Molecular nutrition & food research.*.

[5] Simpson R. U., Hershey S. H., Nibbelink K. A. (2007). Characterization of heart size and blood pressure in the vitamin D receptor knockout mouse. *The Journal of Steroid Biochemistry and Molecular Biology*.

[6] Porto C. M., Silva V. D. L., da Luz J. S. B., Filho B. M., da Silveira V. M. (2018). Association between vitamin D deficiency and heart failure risk in the elderly. *ESC heart failure*.

[7] Sugden J. A., Davies J. I., Witham M. D., Morris A. D., Struthers A. D. (2008). Vitamin D improves endothelial function in patients with type 2 diabetes mellitus and low vitamin D levels. *Diabetic Medicine*.

[8] Zittermann A., Ernst J. B., Prokop S. (2020). A 3 year post-intervention follow-up on mortality in advanced heart failure (EVITA vitamin D supplementation trial). *ESC Heart Failure*.

[9] Musso G., Cassader M., Cohney S. (2016). Fatty liver and chronic kidney disease: novel mechanistic insights and therapeutic opportunities. *Diabetes Care*.

[10] Wortsman J., Matsuoka L. Y., Chen T. C., Lu Z., Holick M. F. (2000). Decreased bioavailability of vitamin D in obesity. *The American Journal of Clinical Nutrition*.

[11] Zoccali C., Curatola G., Panuccio V. (2014). Paricalcitol and endothelial function in chronic kidney disease trial. *Hypertension*.

[12] Tamayo M., Martín-Nunes L., Val-Blasco A. (2020). Beneficial effects of paricalcitol on cardiac dysfunction and remodelling in a model of established heart failure. *British Journal of Pharmacology*.

[13] Sorokina N., O’Donnell J. M., McKinney R. D. (2007). Recruitment of compensatory pathways to sustain oxidative flux with reduced carnitine palmitoyltransferase I activity characterizes inefficiency in energy metabolism in hypertrophied hearts. *Circulation*.

[14] Parra V., Verdejo H. E., Iglewski M. (2014). Insulin stimulates mitochondrial fusion and function in cardiomyocytes via the Akt-mTOR-NF*κ*B-Opa-1 signaling pathway. *Diabetes*.

[15] Zhang L., Jaswal J. S., Ussher J. R. (2013). Cardiac insulin-resistance and decreased mitochondrial energy production precede the development of systolic heart failure after pressure-overload hypertrophy. *Heart Failure*.

[16] Zhou X., Chen J. (2014). Is treatment with trimetazidine beneficial in patients with chronic heart failure?. *PLoS One*.

[17] Lopatin Y., Volgograd State Medical University, Volgograd Regional Cardiology Centre, Volgograd, Russia (2015). Metabolic therapy in heart failure. *Cardiac Failure Review*.

[18] Calton E. K., Keane K. N., Soares M. J. (2015). The potential regulatory role of vitamin D in the bioenergetics of inflammation. *Current Opinion in Clinical Nutrition & Metabolic Care*.

[19] Adela R., Borkar R. M., Mishra N. (2017). Lower serum vitamin D metabolite levels in relation to circulating cytokines/chemokines and metabolic hormones in pregnant women with hypertensive disorders. *Frontiers in Immunology*.

[20] Manna P., Achari A. E., Jain S. K. (2018). 1, 25 (OH) 2-vitamin D 3 upregulates glucose uptake mediated by SIRT1/IRS1/GLUT4 signaling cascade in C2C12 myotubes. *Molecular and Cellular Biochemistry*.

[21] Marcotorchino J., Tourniaire F., Astier J. (2014). Vitamin D protects against diet-induced obesity by enhancing fatty acid oxidation. *The Journal of Nutritional Biochemistry*.

[22] Asemi Z., Hashemi T., Karamali M., Samimi M., Esmaillzadeh A. (2013). Effects of vitamin D supplementation on glucose metabolism, lipid concentrations, inflammation, and oxidative stress in gestational diabetes: a double-blind randomized controlled clinical trial. *The American Journal of Clinical Nutrition*.

[23] Calton E. K., Keane K. N., Soares M. J., Rowlands J., Newsholme P. (2016). Prevailing vitamin D status influences mitochondrial and glycolytic bioenergetics in peripheral blood mononuclear cells obtained from adults. *Redox Biology*.

[24] Peng X., Shang G., Wang W. (2017). Fatty acid oxidation in zebrafish adipose tissue is promoted by 1*α*,25(OH)_2_D_3_. *Cell Reports*.

[25] Alkharfy K. M., Al-Daghri N. M., Ahmed M., Yakout S. M. (2012). Effects of vitamin D treatment on skeletal muscle histology and ultrastructural changes in a rodent model. *Molecules*.

[26] Ricca C., Aillon A., Bergandi L., Alotto D., Castagnoli C., Silvagno F. (2018). Vitamin D receptor is necessary for mitochondrial function and cell health. *International Journal of Molecular Sciences*.

[27] Longoni A., Kolling J., Siebert C. (2017). 1,25-Dihydroxyvitamin D_3_ prevents deleterious effects of homocysteine on mitochondrial function and redox status in heart slices. *Nutrition Research*.

[28] Gambardella J., De Rosa M., Sorriento D. (2018). Parathyroid hormone causes endothelial dysfunction by inducing mitochondrial ROS and specific oxidative signal transduction modifications. *Oxidative Medicine and Cellular Longevity*.

[29] Aleksova A., Ferro F., Gagno G. (2020). Diabetes mellitus and vitamin D deficiency: comparable effect on survival and a deadly association after a myocardial infarction. *Journal of Clinical Medicine*.

[30] Zhang Q., Cheng Y., He M., Li T., Ma Z., Cheng H. (2016). Effect of various doses of vitamin D supplementation on pregnant women with gestational diabetes mellitus: a randomized controlled trial. *Experimental and Therapeutic Medicine*.

[31] Swart K. M., Lips P., Brouwer I. A. (2018). Effects of vitamin D supplementation on markers for cardiovascular disease and type 2 diabetes: an individual participant data meta-analysis of randomized controlled trials. *The American Journal of Clinical Nutrition*.

[32] Parsanathan R., Jain S. K. (2018). Glutathione deficiency induces epigenetic alterations of vitamin D metabolism genes in the liver of high-fat diet–induced type 2 diabetic mice. *Diabetes*.

[33] Lai C. C., Liu C. P., Cheng P. W. (2016). Paricalcitol attenuates cardiac fibrosis and expression of endothelial cell transition markers in isoproterenol-induced cardiomyopathic rats. *Critical Care Medicine*.

[34] Yildirim Y., Yilmaz Z., Kadiroglu A. K. (2016). Mp179 pretreatment with paricalcitol attenuates oxidative stress in renal ischemia reperfusion induced nephropathy in rats. *Nephrology Dialysis Transplantation*.

[35] Wu-Wong J. R. (2009). Potential for vitamin D receptor agonists in the treatment of cardiovascular disease. *British Journal of Pharmacology*.

[36] Panchal S. K., Poudyal H., Iyer A. (2011). High-carbohydrate high-fat diet–induced metabolic syndrome and cardiovascular remodeling in rats. *Journal of Cardiovascular Pharmacology*.

[37] Zhang Y., Sowers J. R., Ren J. (2012). Pathophysiological insights into cardiovascular health in metabolic syndrome,. *Experimental Diabetes Research*.

[38] Zhang Y., Whaley-Connell A. T., Sowers J. R., Ren J. (2018). Autophagy as an emerging target in cardiorenal metabolic disease: from pathophysiology to management. *Pharmacology & Therapeutics*.

[39] Meems L. M., Cannon M. V., Mahmud H. (2012). The vitamin D receptor activator paricalcitol prevents fibrosis and diastolic dysfunction in a murine model of pressure overload. *The Journal of Steroid Biochemistry and Molecular Biology*.

[40] Bae S., Yalamarti B., Ke Q. (2011). Preventing progression of cardiac hypertrophy and development of heart failure by paricalcitol therapy in rats. *Cardiovascular Research*.

[41] Freundlich M., Li Y. C., Quiroz Y. (2014). Paricalcitol downregulates myocardial renin–angiotensin and fibroblast growth factor expression and attenuates cardiac hypertrophy in uremic rats. *American Journal of Hypertension*.

[42] Gong H. P., Tan H. W., Fang N. N. (2009). Impaired left ventricular systolic and diastolic function in patients with metabolic syndrome as assessed by strain and strain rate imaging. *Diabetes Research and Clinical Practice*.

[43] Wu H., Chen L., Xie J. (2016). Periostin expression induced by oxidative stress contributes to myocardial fibrosis in a rat model of high salt-induced hypertension. *Molecular Medicine Reports*.

[44] Repo J. M., Rantala I. S., Honkanen T. T. (2007). Paricalcitol aggravates perivascular fibrosis in rats with renal insufficiency and low calcitriol. *Kidney International*.

[45] Rosca M. G., Tandler B., Hoppel C. L. (2013). Mitochondria in cardiac hypertrophy and heart failure. *Journal of Molecular and Cellular Cardiology*.

[46] Jelenik T., Roden M. (2013). Mitochondrial plasticity in obesity and diabetes mellitus. *Antioxidants & Redox Signaling*.

[47] Sivitz W. I., Yorek M. A. (2010). Mitochondrial dysfunction in diabetes: from molecular mechanisms to functional significance and therapeutic opportunities. *Antioxidants & Redox Signaling*.

[48] Scarpulla R. C. (2011). Metabolic control of mitochondrial biogenesis through the PGC-1 family regulatory network. *Cell Research*.

[49] Savkur R. S., Bramlett K. S., Stayrook K. R., Nagpal S., Burris T. P. (2005). Coactivation of the human vitamin D receptor by the peroxisome proliferator-activated receptor *γ* coactivator-1 *α*. *Molecular Pharmacology*.

[50] Remington S. J. (1992). Structure and mechanism of citrate synthase. *Current Topics in Cellular Regulation*.

[51] Meyer J. N., Leuthner T. C., Luz A. L. (2017). Mitochondrial fusion, fission, and mitochondrial toxicity. *Toxicology*.

[52] Hu L., Ding M., Tang D. (2019). Targeting mitochondrial dynamics by regulating Mfn2 for therapeutic intervention in diabetic cardiomyopathy. *Theranostics*.

